The article "Design of New Power Management Circuit for Light Energy Harvesting System" was retracted in 2016. Reasons: plagiarized text; plagiarized images; false authorship.

# Design of New Power Management Circuit for Light Energy Harvesting System

**DOI:** 10.3390/s16030270

**Published:** 2016-02-23

**Authors:** Issa Jafer, Paul Stack, Kevin MacNamee

**Affiliations:** School of Engineering, University College Cork, Western Road, Cork, Ireland; Paul_Stack@campus.ie (P.S.); Kevin.Macnamee@Campus.ie (K.M.)

**Keywords:** light harvesting, Wireless Sensors Network, maximum power point tracking and boost converter

## Abstract

Nowadays, it can be observed that Wireless Sensors Networks (WSN) are taking increasingly vital roles in many applications, such as building energy monitoring and control, which is the focus of the work in this paper. However, the main challenging issue with adopting WSN technology is the use of power sources such as batteries, which have a limited lifetime. A smart solution that could tackle this problem is using Energy Harvesting technology. The work in this paper will be focused on proposing a new power management design through harvesting indoor light intensity. The new approach is inspired by the use of the Fractional Open Circuit Voltage based Maximum Power Point tracking (MPPT) concept for sub mw Photo Voltaic (PV) cells. The new design adopts two main features: First, it minimizes the power consumed by the power management section; and second, it maximizes the MPPT-converted output voltage and consequently improves the efficiency of the power conversion in the sub mw power level. The new experimentally-tested design showed an improvement of 81% in the efficiency of MPPT conversion using 0.5 mW input power in comparison with the other presented solutions that showed less efficiency with higher input power.

## 1. Introduction

A Wireless Sensor Network (WSN) is a concept that has gradually emerged in the last two decades. One area of greatest potential is in Building Energy Management (BEM) WSN systems [1,2,3]. In the International Energy Outlook, 2011 report issued by the United States Department of Energy, 37% of global energy usage and over 40% of CO_2_ emissions can be attributed to the operation of residential and commercial buildings, as shown in Figure 1 [4]. By monitoring and controlling artificial lighting, temperature, energy consumption, carbon dioxide levels, relative humidity, and airflow, a substantial percentage of energy can be saved [5].

At present, this type of network normally consists of wireless sensor nodes (also known as motes) featuring sensors data processing and communication capability. Recent advances in integrated circuit design and wireless communication research enable these motes to evolve in terms of transmit range, data throughput, processing power, sensor types, and accuracy *etc*. WSN technologies are moving towards further miniaturization [6], smart communication [7,8], and ultra-low energy consumption [9,10].

WSN development is moving towards the target of interconnected small tabs with ubiquitous computing capability. However, one fundamental obstacle to “weave WSN into the fabric of everyday life” is the limited battery lifetime. Due to the limits on the system form factor, the physical size of battery needs to be small, which in turn limits the capacity of the battery.

To effectively prolong the lifetime of WSN systems, energy harvesting technologies have been proposed. Harvesting energy from ambient environments provides a way to not only prolong the system lifetime, but eliminates the need for battery energy storage. In simple terms, it is a process that supplies WSN with small but infinite environmental energy. In this way, WSN lifetime is no longer constrained by the finite local stored energy in the battery but only limited by the lifetime of the energy harvesting module (EHM) and the WSN’s electronic components.

The basic concept of energy harvesting (EH) is a system which converts ambient energy into electricity, as shown schematically in Figure 2. However, although electricity is harvested from the ambient environment, without output power management, it cannot be used in this unconditioned form to power a wireless sensor node. Without an energy storage unit, any glitch in the ambient energy source will lead to “mote” power failure. Furthermore, without input power management on the energy harvesting unit, the energy conversion is not optimized and cannot deliver energy with high efficiency and reliability.

The focus of this paper is mainly on the development of power management circuits for indoor light energy harvesting. Light energy can be considered as the most ubiquitous ambient energy source, although it generally has low light intensity (300 lux–500 lux) as opposed to high power density outdoor lighting (>2000 lux for a cloudy day [11]).

Maximum power point tracking (MPPT) technologies have often been used for solar power systems with output power higher than 100 mW [12,13]. By implementing switching regulator-based MPPT techniques, the EHM will operate near its theoretical maximum power point and generates power close to its highest conversion efficiency. One major challenge in energy harvesting systems is how to implement this type of input power management circuit with minimum power consumption overhead. The conventional methods of MPPT cannot be directly adopted because their power consumption is beyond the power budget of the small EH system, *i.e.*, 1 mW or even lower. In this paper, a new method has been proposed in order to perform Ultra-low Power (sub 1 mW) MPPT. In addition to the MPPT issue, the energy harvesters often generate lower voltage than conventional power supplies such as batteries. Once the optimized output power of energy harvesting unit (EHU) is harvested, it is necessary to store the harvested energy using energy storage units (ESU). ESU such as super-capacitor, thin film battery and commercial off-the-shelf rechargeable batteries are considered in this work. Based on the nature of these ESUs, the related charge/discharge control circuits, such as controlled-start circuits and output voltage regulation circuits, for ESU power management are proposed. Figure 3 illustrates the proposed power management structure for the energy harvesting system.

In terms of prototype development, the objective of this work is to design a continuous and maintenance-free power management system for an energy harvester module in low duty cycle WSN applications. With a credit card form factor (less than 80 mm × 50 mm), the device should be able to supply the power consumption of WSN with regulated power from a typical building environment. The average conversion efficiency of the power management circuits should be higher than previous state-of-the-art circuits and the prototypes should be required to have a minimal lifetime of 10 years. The proposed power management module consisting of a PV (Photo Voltaic) cell designated for indoor light energy harvesting, low power control logic circuits, discrete components-based switching regulator, specific control scheme, and an energy storage unit with controlled-starting circuit will be introduced in the next section to achieve these two design goals. The complete energy harvester for a Wireless Zigbee mote block diagram is shown in Figure 4.

This paper is organized as follows: Section 2 introduces the related work overview and highlights the main contributions to the work presented in this paper. The experimental setup of the presented power management system using three main stages that adopt the concept of synchronized boost converter-based MPPT is described in Section 3. Section 4 presents the simulation and experimental results, and final conclusions are drawn in Section 5.

## 2. Related Work and Contribution

This section introduces a detailed overview of energy harvesting technologies for WSN applications that have been developed in the past with a focus on power management circuits and simulation. Farhan *et al.* introduced a pulse frequency modulated (PFM) power management unit with maximum power point tracking capability. The MPPT method utilizes the mote micro-controller to adjust the frequency and duty cycle to operate near the maximum power point condition [14]. This method is a very typical example of MPPT circuit design. It adopts a “perturb and observe” method which requires a micro-controller to constantly monitor and adjust the frequency of the PFM control signal on the buck converter. This significantly increases the system cost and complexity. The power consumption of the current sensor and the ADC of the microcontroller are far beyond the harvestable power from indoor light. Although the system can obtain 80% efficiency when it operates with 20 mW input power, the adoption of this MPPT approach for indoor light energy harvesting is impractical. The less than 1 mW harvestable power in indoor conditions obviously cannot operate the 5 mW MPPT circuitry.

In Park and Chou’s paper [15], a different sensor method is proposed for its lower power consumption. Instead of the commonly used current sensor, a light intensity sensor is used in this case to monitor light level and simulate the power output instead of current sensing. The micro-controller is programmed with a lookup table with relevant control modes in different light intensities. When the light condition varies, the microcontroller changes the control mode in order to maximize the harvested energy. The power consumption of this MPPT circuit is approximately 2 mW, based on the efficiency calculation given in the paper.

Brunelli *et al.* presented an analog comparator controlled PWM buck converter based on the FVOC MPPT design principle without using complicated DSP or micro-controller in [16]. The adoption of analog comparator based control circuits significantly reduced the power consumption in the MPPT circuits by one order of magnitude from 10–100 mW to 1–10 mW level. Although the conversion efficiency of 80% achieved at 10 mW is similar to that in previous work which utilized the Perturb and Observe method (84%) at 10 mW [17], it shows promise of a low power consumption solution to tracking MPP.

This group also published [18,19,20] from the perspectives of simulation and components selection improvement of this method. This work analyzed the power loss in an MPPT circuit and the impacts on the system conversion efficiency for 10–50 mW input power applications. The power loss is mainly attributed to the switching loss of the converter, conduction loss associated with the inductor, super-capacitors, and diode forward voltage drop in the buck converter circuit. In [21] Brunelli *et al.* presented a system that is similar to the design described in this paper. A 50 F supercapacitor is used as the energy storage. The PWM-controlled MPPT circuit implements the fractional open circuit voltage method. The carefully simulated and implemented MPPT sub-system only requires mW-level power consumption. However, due to the inherent relatively high power consumption of the PWM circuits, potential for further MPPT circuit power consumption reduction is limited.

In fact, Brunelli and Benini suggested that due to the power consumption in the MPPT, small PV cells are impractical to use in the MPPT to improve conversion efficiency, and an alternative method should be adopted instead. In [20], a semi-MPPT design with a two voltage comparator was adopted. The main drawbacks of this design are: Firstly, it cannot power the mote when no direct light is available. Once the capacitor voltage drops lower than threshold voltage, with no input power charging the capacitor, the mote cannot operate; Secondly, the output voltage of this design is not a regulated voltage. The WSN mote operation time and frequency are not programmed by WSN mote, but instead rely on the input light and capacitor size. This simple “semi-MPPT” method operates with high efficiency at 90% in indoor conditions. However, for most building applications which require a constant duty cycle, e.g., WSN mote programmed to operate every 1 min, this method is not suitable due to its variable charge/discharge time.

Tan’s work [22] shows that the low frequency low duty cycle PWM control signal and related DC-DC converter design leads to small power losses in the MPPT switching regulator. However, the complicated Perturb and Observe MPPT control logic in [22] still consumes considerable power (0.36 mW) and requires both current and voltage sensors to monitor the solar cell. FVOC ultra-low power analog comparator control logics from Brunelli’s work [16] shows it is possible to achieve low power consumption from this simple and low power control logic. However, the high frequency high duty cycle operation of the DC-DC converter used in [16] limits its efficiency.

Tan and Panda also applied the low frequency low duty cycle PWM control method to indoor light and thermal hybrid energy harvesting with a voltage sensor-based MPPT control logic in an attempt to resolve the aforementioned control logic power consumption issue as reported in [23]. The main drawbacks of this MPPT method are: (1) Although it reduces the power consumption of the logic circuits, the 0.135 mW power consumption is still considerable for sub-mW MPPT; (2) In this work, in order to acquire the open circuit voltage of the solar cell and thermoelectric generator, a light sensor and temperature sensor are used to generate the light/temperature data. The data is then processed by the micro-controller and compared to the pre-stored look-up table based on the measurement of the selected type of solar cell and thermoelectric generator. An algorithm has to be created to adjust the PWM for each type of solar cell in order to respond to the reference voltage; (3) The system cost and complexity is very high—the utilization of an additional 16-bit micro-controller in order to control a maximum power point tracker has only been seen in kW/MW-level solar power plant applications; (4) Although not clarified in the paper, it also potentially poses a self-start issue for the power supply control logics.

Alippi and Galperti [24] introduced a low-power-based MPPT design using an adaptive tracking power converter system. The system is also using an MCU to implement the control algorithm resulting in a low efficiency figure of 26.4%, which means that the system needs further improvements. These findings lead to the aim in this paper to combine the highlighted advantages of each approach in order to achieve ultra-low power consumption MPPT solution. Our approach is to avoid the use of the MCU and utilize the fractional open circuit voltage (FVOC) approach and adopt an analog comparator-based control logic design. Synchronized switching was introduced in the boost converter of the sub-mW MPPT instead of the diode rectification to reduce potential conduction power losses. In addition, a new controlled start circuit was designed to provide sustainable and stable regulated power for long-term wireless sensors nodes deployment in a building environment where indoor light intensity is low and variable.

## 3. Experimental Section

### 3.1. Indoor Light Photovoltaic Cell

Commercial off-the-shelf (COTS) PV cells and home-designed PV cells have been tested with various light sources and light intensity conditions. The halogen illumination is generated from the Euromex EK-1 light illuminator. The low light intensity measurements are conducted with a fluorescent lamp. The intensity of the light was measured with a light meter in an integrating sphere (in order to obtain an evenly-distributed light scattering on the sample and light meter). Figure 5 shows the testing layout before the samples are placed onto the integrating sphere sample holder.

### 3.2. Maximum Power Point Tracking

PV cells have I-V (current-voltage) characteristics similar to a voltage controlled current source [13]. As introduced in literature reviews, similar to the concept introduced in [13,25], the FVOC method is adopted in this design. The simple computation and low power consumption make this MPPT method suitable for small-scale PV devices. The MPPT method in this work differentiates from previous literatures in six aspects:

1. Low-frequency MPPT is adopted in this work in order to reduce the switching loss on the MOSFET.
2. Instead of operating in the converter continuous conduction mode, this MPPT converter operates in discontinuous conduction mode with lower inductor current. This is beneficial for reducing certain conduction losses on Equivalent Series resistance (ESR).
3. The MPPT Pulse Width Modulation (PWM) control signal is generated from the analog comparator instead of the signal generator circuit in order to reduce the MPPT control logic power consumption.
4. A pilot PV cell (Sanyo AM1417) made from the same technology as the main PV cell (Sanyo AM1815/16) is used as the voltage reference. Instead of disconnecting the PV cell to measure the VOC, the pilot PV cell provides a reference VOC which is proportional to the open circuit voltage of the main PV cell. This method further reduces the complexity and power consumption of the MPPT controller.
5. Modelling and optimization is for sub 1 mW input power. The key parameter for power loss analysis including inductor current and the MPPT upper/lower voltage thresholds are optimized towards higher conversion efficiency.
6. The efficiency evaluations are based on capacitive load instead of resistive load. This evaluation method can reflect the energy harvester efficiency more accurately in real-world deployment scenario.

#### Synchronized Boost Converter MPPT

In the power loss analysis of the buck converter MPPT circuit [25,26,27], one obvious discovery is that the body diode forward voltage drop contributes greatly to the total power loss. Synchronized rectifier switching regulation is frequently used to reduce the power loss in the diode forward voltage drop. The conventional synchronized rectification (SR) requires the use of specific control FET with a Schottky diode, monitoring the inductor current by inserting a 10–30 mΩ sense resistor in series with the inductor and auxiliary control system. The control system operates the two MOSFETs individually and often uses certain algorithms to maintain a short but compulsory “dead time” and ensures “break-before-make”. For the energy harvesting system, such complex power management is difficult to achieve with a small power budget.

A new synchronized rectification method is introduced in this work to operate SR with pre-calculated dead time without complex control circuits and Schottky diodes offering a very low conduction loss.

The schematic of the synchronous boost converter based MPPT is shown in Figure 6. The MPPT consists of two main building blocks. (1) Comparator based MPPT controller; (2) synchronous boost converter. The boost converter is controlled by PWM signals generated from the ultra-low power comparators. A secondary PV cell is used to obtain a reference open-circuit voltage V_PV_Ref_ to set the theoretical V_MPP_.

### 3.3. Controlled-Start Circuit for ESU

The method for controlled-start circuit design is to build a circuit to prevent the input power management switching regulator and output power regulator from starting up before they reach the required voltage. It is essential to obtain a self-start circuit to achieve two targets:

1. The controlled-start circuits provide logic control to switch on the enable pins of the switching regulators only when the input voltages exceed the switching regulator start-up voltage.
2. The controlled-start circuits should provide a stable voltage supply for the output power regulator to continuously operate the output regulator until the ESU reaches minimum operational voltage.

The controlled-start circuit is introduced in Figure 7. This sub-system is largely separated from the rest of the energy harvester to ensure its reliability. A secondary PV cell is used in this self-start circuit design to function as an individual power supply. REF3312 is Texas Instruments voltage reference IC with 1.25 V output reference voltage (when input voltage is higher than 1.5 V). The components values of the self-start circuit are shown in Table 1, large resistors are chosen for low leakage current through the voltage divider arrays.

### 3.4. Energy Harvesting WSN Case Study

A case study was conducted from 14 March 2015 to 2 April 2015 (more than 2 weeks) to test the operation of an energy harvesting powered wireless sensor node in typical office conditions. COT Zigbee wireless motes were used for this purpose [28]. The test location was conducted in my office room (typical office environment). There is no direct sunlight at this location. The nearest window (northeast facing) is 5 m away. The light source is provided by multiple groups of overhead fluorescent lamps. The configuration of this typical office environment test is illustrated in Figure 8.

## 4. Results and Discussion

### 4.1. Testing of Maximum Power Point Tracking

The I-V characteristics of the PV cell in an indoor condition illustrate that a 10% MPPT error illustrated in Figure 9 only leads to <5% power loss due to FVOC-based MPPT inaccuracy. Although the FVOC MPPT method has inferior dynamic tracking capability and tracking accuracy when compared to other methods, for low light intensity conditions such parameters are less important. Reducing power consumption in the MPPT is the design priority for this small PV energy harvester.

#### Simulation Results of Boost Converter MPPT

A SPICE model is created to simulate the boost converter MPPT. The captured simulation results show two cycles of the power tracking process in Figure 10. Hysteresis is adopted in the design to switch on transistor SW1 when input capacitor voltage (PV cell voltage) is higher than *V_MPP_ + V_hyst1_*. The input capacitor is then discharged whilst the inductor L is charged with variable current *I_L_(t).* Once the capacitor voltage drops to *V_MPP_* − *V_hyst1_*, the SW1 is turned off due to the hysteresis, the ON stage time is from *t*_0_ to *t*_1_.

It is worth noting that the charging process in the simulation adopts small output capacitors in order to accelerate the charging speed and better illustrate the results. In actual cases, the time between t_2_ and t_3_ is 1–2 orders of magnitude longer than this simulation. SW2 is switched on when PV cell voltage is within *V_MPP_ + V_hyst2_* and *V_MPP_* − *V_hyst2_*. The hysteresis voltage *V_hyst2_* is larger than the hysteresis for SW1 *V_hyst1_*.

SW3 is controlled with a voltage comparator without hysteresis as shown in Figure 10. SW3 is only switched on when PV cell voltage drops to *V_MPP_* − *V_hyst1_* − *V_deadtime_*. The additional voltage difference *V_deadtime_* ensures SW3 only switches on after the SW2 is completely switched off. Thus, in a short period t_deadtime_ (known as dead-time) both SW1 and SW3 are switched off to avoid shorting the output of the super-capacitor reversely through SW1. After SW3 is turned on, the energy stored in the inductor, L, is discharged into the output capacitor, *C_OUT_*, in this phase. The hysteresis can be easily adjusted by scaling the resistors in the voltage divider to amend the MPPT accuracy and frequency.

The adoption of the two switches SW2 and SW3 in series provides a means to better control the on/off time and dead-time with simple and low power comparator logics. SW1-3 performs a synchronous rectification without output switch drive. Similar to the hysteresis adjustment, the dead-time can then be changed with the resistance of the comparator voltage divider. The power loss on the diode forward voltage drop is entirely eliminated in the design. As a result, the power conversion efficiency is improved. In order to assess the concept and optimize the MPPT design, a SPICE simulation for power loss analysis is created with its equivalent schematics, shown in Figure 11. The power loss model describes the three phases of the energy conversion.

The converter “on-stage” when SW1 is switched on between t_0_ and t_1_ is shown in Figure 11a. The converter “off-stage” where SW1 is off, SW2 and SW3 are on between t_1_ and t_2_ is shown in Figure 11b. The “idle-stage” when all transistors are switched off, while the input capacitor is charged from the PV cell between t_2_ and t_3_ is also shown in Figure 11b.

The power loss analysis in the following paragraphs is based on the equivalent circuit analysis in Figure 11 and the simulation results shown in Figure 10. The power loss in the MPPT circuits consists of conduction loss, control IC power consumption, and switching loss. The <1 mW low input PV cell power can only charge the input capacitor at a relatively low speed, the magnitude of the cycle time *T_s_* is of the order of 10 ms, the boost converter operating at a frequency of less than 1 KHz. Due to the low frequency and the low current nature of the circuits, the switching loss is negligible. The main energy losses are due to conduction loss *E_cond_*, MPPT error *E_error_* and control IC power consumption *E_ctrl_*.

(1) *E_loss_ = E_cond_ + E_error_ + E_ctrl_*

The power consumption of control IC is near constant and mainly relies on the COTS comparator IC. The main variable in the power analysis is the conduction loss in the inductor, on-resistance of transistors, and internal resistance of capacitors. As illustrated in Figure 11, the boost converter operates in discontinuous conduction mode (DCM mode). The power loss analysis is then divided into three stages: On-stage, off-stage, and idle-stage.

**On-Stage:** At time *t*_0_, the PV cell voltage, also the input capacitor voltage, *V_PV_* reaches the upper voltage limit of the pre-set MPPT hysteresis *V_MPP_ + V_hyst1_*. SW1 is then switched on, the input capacitor transfers the stored energy into the inductor and the PV cell also charges the inductor in this stage. The voltage behaviour is shown in Equation below:

(2) $$V_{L}=L\frac{di_{L,on}\left(t\right)}{dt}=V_{pv}\left(t\right)-\left(R_{L}+R_{ds,on}\right)\cdot I_{L,on}\left(t\right)$$

The inductor current, the main impact factor of the power loss, is shown in Equation (3). The inductor current increases until time t_1_ and dissipates power on inductor internal resistance and on resistance of the transistor.

(3) $$\begin{array}{cc} \frac{1}{2}I_{Lmax}^{2}L+\;\int_{0}^{Ton} & I_{L,on}^{2}\left(t\right)\;\cdot \;\left(R_{L}+R_{ds,on}+\;R_{Cin\;}\right)dt\\ & =\frac{1}{2}\;C_{in}\;\left[{\left(V_{mpp}+V_{hyst1}\right)}^{2}-{\left(V_{mpp}-V_{hyst1}\right)}^{2}\right]+\;P_{pv\;}\cdot T_{on} \end{array}$$

The on stage time T_on_ is mainly determined by the hysteresis and input capacitor. Due to the near linear increases of the inductor current (also proved in the SPICE simulation), the inductor current can be approximated by the following equation,

(4) $$I_{L,on}\left(t\right)=\frac{I_{L\;max}}{T_{on}}\;\cdot \;t$$

With the presumed linear correlation between inductor current *I_L,on_* and time t, the energy transfer during on stage in Equation (3) is changed into,

(5) $$\frac{1}{2}\;I_{Lmax}^{2}\;L+\;\frac{1}{3}\;I_{Lmax}^{2}\;\left(R_{L}+R_{ds,on}+\;R_{Cin\;}\right)T_{on}=2\;C_{in}\;V_{hyst1}\;V_{mpp}\;+\;P_{pv\;}\cdot \;T_{on}$$

In the input capacitor, the voltage decreases from *V_MPP_ + V_hyst1_* to *V_MPP_ − V_hyst1_*, the voltage change can be expressed in the following equation,

(6) $$V_{mpp}-V_{hyst1}=V_{mpp}+V_{hyst1}-\frac{1}{C_{in}}\int_{0}^{Ton}I_{L,on}^{2}\left(t\right)dt$$

The equation can be further simplified into,

(7) $$2V_{hyst1}=\frac{1}{2}\frac{I_{L\;max}T_{on}}{C_{in}}$$

By combining Equations (5) and (7), inductor maximum current *I_Lmax_* can be derived in the following equation,

(8) $$\frac{1}{2}\;I_{Lmax}^{3}\;L+\;\frac{4}{3}\;I_{Lmax}^{2}\;\left(R_{L}+R_{ds,on}+\;R_{Cin\;}\right)\cdot V_{hyst1}\cdot \;C_{in}-2\;V_{hyst1}\cdot \;C_{in}\cdot V_{mpp}\cdot I_{L\;max}-4P_{pv\;}V_{hyst1}\cdot \;C_{in}=0$$

Once *I_Lmax_* is known, the “on” stage time *T_on_* can be calculated using the following equation derived from Equation (7),

(9) $$T_{on}=\frac{4V_{hyst1}C_{in}}{I_{L\;max}}$$

Once the input capacitor voltage (also the PV cell voltage) drops to *V_mpp_Vhyst1_*, switch SW1 is turned on. The MPPT converter enters the “OFF” stage.

**OFF-Stage:** From t_1_–t_2_, the switches SW2 and SW3 are switched on, the energy accumulated in the inductor and input capacitor is discharged into the ESU. Based on the SPICE simulation, it is obvious that the MPPT converter is operating in discontinues conduction mode. In the off-stage, the inductor current decreases from *I_Lmax_–*zero.

The voltage in input capacitor C_in_ further decreases in this stage from *V_mpp_ − V_hyst1_* to *V_mpp_ − V_hyst2_* as shown in the SPICE simulation. Hysteresis voltage *V_hyst2_* is also set by the comparator resistor array. The voltage change in the input capacitor can be used to express the relationship between the off stage time *T_off_*, inductor current *I_off_ (t)* and the hysteresis voltages,

(10) $$V_{mpp}-V_{hyst2}=V_{mpp}-V_{hyst1}-\frac{1}{C_{in}}\int_{0}^{Toff}I_{off}^{2}\left(t\right)dt$$

Assuming a linear correlation between “off” stage time and inductor current,

(11) $$I_{L,off}\left(t\right)=I_{L\;max}\left(1-\frac{t}{T_{off}}\right)$$

Considering the linear correlation, the Equation (10) becomes,

(12) $$V_{hyst2}-V_{hyst1}=\frac{1}{2}\frac{I_{Lmax\;}T_{off}}{C_{in}}$$

Since maximum inductor current *I_Lmax_* is known, *T_off_* is directly determined by hysteresis voltages and the input capacitor. In this stage, since the diode is replaced by synchronous switches, the *I_L_V_fd_* diode forward voltage drop power loss is replaced by the switch on resistance conduction loss *I_L_^2^*·*R*.

The equivalent resistance in the converter during this stage *R_off_* is comprised of ESR of inductor *R_L_*, on resistance of SW2 and SW3 *R_ds,on_*, input capacitor ESR *R_cin_* and super-capacitor ESR *R_cap_*,

(13) $$R_{off}=R_{L}+2\cdot \;R_{ds,on}+R_{cin}+R_{cap}$$

The energy transfer from the input capacitor and inductor to the super-capacitor in this stage can be described as,

(14) $$\begin{array}{cc} \frac{1}{2}I_{Lmax}^{2}L+\;\frac{1}{2}C_{in} & \left[{\left(V_{mpp}-V_{hyst1}\right)}^{2}-{\left(V_{mpp}-V_{hyst2}\right)}^{2}\right]\\ & =\int_{t1}^{t2}I_{L,off}^{2}(t)\;\cdot \;R_{off}dt\\ & +\frac{1}{2}\;C_{cap}\;\left[{\left(V_{cap}+\frac{1}{C_{cap}}\int_{t1}^{t2}I_{L,off}^{2}(t)dt\right)}^{2}-V_{cap}^{2}\right] \end{array}$$

With a linearly decreasing inductor current, the energy transfer in Equation (14) becomes,

(15) $$\begin{array}{cc} \frac{1}{2}I_{Lmax}^{2}L+\;\frac{1}{2}C_{in} & \left[{\left(V_{mpp}-V_{hyst1}\right)}^{2}-{\left(V_{mpp}-V_{hyst2}\right)}^{2}\right]\\ & =\frac{1}{3}\;I_{Lmax}^{2}\cdot \;R_{off\;}\cdot T_{off}+\frac{1}{2}\;C_{cap}\;\left[{\left(V_{cap}+\frac{I_{Lmax}\cdot T_{off}}{2C_{cap}}\right)}^{2}-V_{cap}^{2}\right] \end{array}$$

In the implementation, the comparator which controls SW3 is carefully adjusted to include a short deadtime in order to avoid SW1, SW2 and SW3 simultaneously conducting current.

Comparing with the buck converter which adopts a rectifier diode [22,23] instead of synchronous switches, the power loss is reduced in this configuration. The detailed power loss analysis is given in Table 2.

**Idle-Stage:** From the time *t_2_*–*t_3_* the MPPT circuit enters an idle stage, SW1, SW2, and SW3 are switched off during this stage, and the input capacitor voltage is charged from the lower hysteresis threshold to the upper threshold. In this work, the input current *I_PV_* is one–two orders of magnitude lower than the inductor current. The conduction power loss in this phase is negligible.

### 4.2. Testing of Controlled-Start Circuit

The test results of the controlled-start circuit are shown in Figure 12. The measurement is conducted with a Pico Technology data logger ADC-11/12. The self-start circuit is firstly placed in 0 lux light intensity when the ESU voltage *V_ESU_* is close to the output regulator minimal operating voltage. *V_EHU_* drops below the voltage threshold at *t_0_*. Both the power supply bus voltage *V_cc_* and the system output voltage *V_wsn_* drop to near zero volts at *t_0_*. A fluorescent light source with 500 lux light intensity is switched on at time *t_1_*. The small input capacitor *C_1_* is then charged towards the required 1.5 V. The minimal light intensity required for the start-up is only 150 lux with the 3.5 cm^2^ secondary PV cell (10 W). When *V_cc_* is close to 1.2 V, it activates the voltage reference and control comparators at *t_2_*. The power management module circuit is then activated by comparator1 (Comp1) and the ESU starts to charge. The ESU is charged to 0.9 V, the minimal start-up voltage preset by the voltage divider, at *t_3_*. Comparator 2 (Comp2) switches on the output regulator enable pin and system output recovers to a regulated *V_wsn_*. The system output voltage *V_wsn_* also starts to function as the voltage supply *V_cc_* gets stable at *t_3_*. The controlled start procedure completes at *t_3_*.

### 4.3. Energy Harvester Implementation

Two types of energy harvesters are designed and implemented. Prototype I implements the MPPT method proposed in Section 3.2 and Prototype II is designed without MPPT optimization (for result comparison and verification purposes). The control logics of MPPT are implemented with two Maxim MAX934 ultra-low power comparators. The power consumption of the control logics during MPPT and ESU charge/discharge is measured at 29 µW. The transistors adopted in this design are Vishay SiB914DK with 0.28 Ω on resistance at 1.5 V Vgs and gate capacitance at 68 pF.

The inductance of the MPPT inductor is 1 mH with equivalent series resistance of 6 Ω. The input capacitor is 140 µF with a 10 mΩ ESR. The output capacitor is a Maxwell 2.5 F super-capacitor with maximum voltage rating at 5 V. The super-capacitor has an internal DC resistance around 2 Ω.

The output voltage regulator is a Texas Instruments TPS61221 boost converter with a minimum input voltage threshold at 0.7 V. The resistance of the voltage divider resistors is between 0.5 MΩ and 10 MΩ. The high resistance reduces the conduction loss in the dividers. The power management system is implemented on a 39 mm × 30 mm PCB. The device is packaged with a polymer case printed by a 3D printer. The Sanyo amorphous silicon-based PV cell has a form factor of 55 mm × 40 mm. The overall device dimension is 88 mm × 60 mm, slightly larger than a standard credit card. The prototype is shown in Figure 13.

The MPPT operation is shown in the captured oscilloscope waveform in Figure 14. The test is conducted under 500 lux fluorescent lighting conditions. Direct comparison was made to evaluate the performance difference between the two prototypes illustrating the charging performance at 500 lux within a time period of 100 s. Within this period of time, a 30 mF super-capacitor is charged to 2.1 V with the proposed MPPT method and only 0.95 V without MPPT. The results clearly show that the charging performance is improved by adopting MPPT for the low power PV cell.

The energy conversion efficiency is calculated by using the Equation below.

(16) $$\gamma_{conv}=\frac{C_{cap}\cdot \left(V_{C1}^{2}-V_{C0}^{2}\right)}{2\cdot P_{PV}\cdot T_{charge}}\;\cdot 100\%$$

By using this proposed MPPT method, the input current and voltage variations are reduced, thus average current and voltage are used to calculate the input PV energy. In this implementation, the average leakage current of the 2.5 F super-capacitor is approximately 25 µA in a 24 h measurement. The conversion efficiency and the harvested power are shown in Figure 15.

In a typical office environment with light intensity at 480 lux^3^ (fluorescent), the theoretical maximum output power of this PV cell is approximately 490 µW. The implemented EH device harvests 395 µW in this condition and the energy conversion efficiency is 80.5%.

Table 3 shows the comparison of efficiency among various maximum power point tracking circuits against their power levels. The measured conversion efficiency of 80.5% is the current state of the art in terms of sub 1 mW MPPT circuits.

### 4.4. Results of Using the New Developed MPPT in WSN Case Study

The lighting condition is within the range of 0 lux (night) to maximum 600 lux (day). A simulated light intensity is also created using developed Matlab model to study the system performance when the light intensity measurement is not available. The measured and simulated light intensity during the 14 days experiments are shown in Figure 16.

The simulation of the office light intensity is shown in the green curve. The simulation light intensity is 300 lux for 4 h, 450 lux for 8 h and 0 lux during the night. The overall product of lux and time is 4800 lux × hour in the simulation, whilst the measured light intensity in one day is also approximately 4800 lux × hour. In the measured light intensity results, the northeast facing window contributes to some of the light intensity and was captured by the light sensor. The average light intensity during the daytime is measured at 410 lux. The weekday and weekend light intensity are also different due to the usage profile. For example, at the 144-hour mark, the light is measured during the weekend. The light intensity only increased to 520 lux at 2 p.m. when the light is turned on, while the light is normally turned on around 8–9 a.m. during weekdays.

The EH device is tested with a Pico Tech Picolog data acquisition module Picolog-1206. It is capable of recording 3 million data sets (recording data for 33 days with 1 second resolution). The indoor light energy harvesting module adopts a Sanyo AM18 series PV cell with an active area of 38 cm^2^ (AM1815). The MPPT circuit is based on the synchronized boost converter design introduced in the previous sections. The output voltage regulator is based on TI TPS61220 converter and the energy storage unit is a Maxwell PowerStor super-capacitor with a 5.0 V voltage rating and 2.5 F capacitance. The ESU voltage is measured for 340 h (nearly 14 days) and presented in Figure 17.

Two simulation results are also presented in this figure. The black line indicates the measured ESU voltage. The blue line indicates the ESU voltage simulation with measured input light intensity, whilst the red line indicates the ESU voltage simulation with simulated input light intensity (300/450 lux at morning-evening/mid-day).

The red bar (shadow area) illustrates the measured light intensity, whilst the blue bar illustrates the simulated light intensity. The results show the mote operating for more than 14 days without power failure when it was solely powered from indoor light with the energy harvesting module designed in this work. The ESU obtained a maximum voltage of 5.1 V (2% higher than the super-capacitor voltage rating) and a minimum voltage of 0.83 V. In the entire deployment, the voltage output of the energy harvester is always measured at 3.3 V with a variation of less than 5%. In this experiment, the energy stored in the ESU accumulated over time and was always higher than the minimum operational voltage threshold in the entire deployment.

Both the measured light intensity and the typical office light intensity simulations show high consistency with the measurement results from the gathered deployment data.

### 4.5. WSN Comparative Study

Light energy-powered WSN system design is an area of ongoing active research interest. Several light energy harvesting systems for WSN have been developed and published in the past. This section gives an overview of some of these systems’ main features in comparison with our presented design.

“Helimote” presented in [30] is one of the first proposed light energy harvesting powered WSN systems. It features a simple outdoor solar panel powered mote system design, directly connecting the solar cell to the energy storage. Energy storage in Helimote is achieved using NiMH rechargeable batteries. The power management lacks an MPPT function, and can only charge the battery when the solar panel output voltage is 0.7 V higher than the battery voltage.

On the other hand, “Prometheus”, presented by Jiang, Polastre, and Culler [31] uses a design similar to Helimote, but it features hybrid energy storage: a combination of an Li-Polymer rechargeable battery and a 22 F supercapacitor. A certain control logic is used to charge the battery from the supercapacitor when the latter is fully charged *versus* directly feeding the battery to the load when the supercapacitor voltage is lower than a defined threshold voltage. This method prolongs the battery lifetime. Similar to the Helimote, it also lacks an MPPT function and requires a high charging voltage.

“Everlast”, presented by Simjee and Chou in [18] implements a design with the elimination of the rechargeable battery. The energy storage element is a 100 F supercapacitor. The Everlast design employs an MPPT algorithm running on the mote’s microcontroller. The MPPT is accurate and operates at a high speed. However, this MPPT method requires a much higher power level from the PV cells and is not a suitable choice for indoor light energy harvesting.

The three light energy harvesting systems discussed above are only suitable for operation in outdoor conditions. The system power consumption and output power of the PV cells are well above the 100 mW level.

In [32] a solar-powered mote system called “Ambimax” was proposed by Park and Chou, uses multiple power sources including solar energy and wind energy. The power sources were managed by a common power conditioning unit. Ambimax automatically tracks the maximum power point without using the microcontroller of the WSN. The energy storage in this system is a supercapacitor and Li-Polymer battery combination. Similar to Prometheus, the system lifetime of this design would also be limited by the battery lifetime. The MPPT subsystem requires a current consumption in the mA range, which is more than an order of magnitude higher than the power consumption of our proposed system.

## 5. Conclusions

In this paper, the concept of using the fractional voltage open circuit (FVOC) method in the sub 1 mW MPPT design for its superior ultra-low power consumption was proved to be feasible, and the implementation is suitable for WSN applications.

With MPPT efficiency as high as 79.6% at 0.9 mW, the buck converter-based MPPT prototype can provide a stable power supply when the input light intensity is only 245 lux. It was concluded that by replacing the high position diode by a synchronized switch and modifying the structure to boost topology, the boost converter-based FVOC MPPT method further reduces the power loss in the MPPT converter. It achieves power gain from input power as low as 80 µW (120–130 lux, credit card sized COT PV cells). With this MPPT design, the energy harvester prototype obtains 81% efficiency at 0.5 mW. This conversion efficiency is higher than previous state-of-the-art [27] that reported 59% in similar condition.

The presented credit card-sized indoor photovoltaic energy harvester supplies 0.2 mW–0.4 mW regulated power to the WSN mote when the solar cell is under 300–500 lux indoor light. This generated power is sufficient for low duty cycle (0.1% or less) using the selected WSN mote. It met the final target of long-term WSN power autonomous operation in a typical office/residential building environment.

## Figures and Tables

**Figure 1:** Global Energy Consumption in terms of U.S. Dollars in 2011 [4].

**Figure 2:** Simple Energy Harvester-Powered WSN (Wireless Sensors Networks).

**Figure 3:** Power Management for Energy Harvesting Systems.

**Figure 4:** Indoor Light Energy Harvester for WSN System Block Diagram.

**Figure 5:** PV (Photo Voltaic) cell illumination tests: (**a**) Samples tests setup; (**b**) Integrating sphere with halogen lamp light source.

**Figure 6:** Schematics of Maximum Power Point Tracking.

**Figure 7:** PV Cell Energy Harvester Self-Start Circuits Schematics.

**Figure 8:** EH powered WSN Deployment Case Study.

**Figure 9:** Measured I-V Characterizations and MPPT error (100–500 lux).

**Figure 10:** Converter SPICE simulation and control signals of SW1, SW2 and SW3.

**Figure 11:** (**a**) On-stage (*t*_0_ − *t*_1_) equivalent circuit (**b**) OFF-stage (*t*_1_ − *t*_2_) equivalent circuit and Idle-stage (*t*_2_ − *t*_3_) equivalent circuit.

**Figure 12:** Screen Capture of Start-up Process in a PV Cell Energy Harvester Based on Controlled-start Circuit (measured with Pico Tech Data Logger).

**Figure 13:** Picture of indoor light EH (energy harvesting)-powered WSN prototype.

**Figure 14:** Boost Converter MPPT Results (Oscilloscope screen capture): (**a**) MPPT tracking PV cell voltage and charging current waveforms; CH1: MPPT Voltage: 200 mV per vertical division. CH2: Inductor Current Measurement using 8 Ω Shunt Resistor with 10× Amplification: voltage-current ratio 80:1. Horizontal: time: 100 ms per division; (**b**) Comparison Charging Super-capacitor with/without MPPT; CH1 and CH2:500 mV per vertical division. Horizontal: time: 10 s per division.

**Figure 15:** MPPT conversion efficiency in sub 1 mW power conditions (100–1000 µW).

**Figure 16:** Light intensity measurement and simulation.

**Figure 17:** EH Powered WSN Deployment Measurement Results.

**Table 1:** Components Parameters of Self-Start Circuit.

R_1_ = 1.5 MΩ	R_2_ = 2 MΩ	R_3_ = 1 MΩ
R_4_ = 1 MΩ	R_5_ = 5.1 MΩ	R_6_ = 310 KΩ
R_7_ = 710 KΩ	R_8_ = 1 MΩ	R_9_ = 1 MΩ
R_10_ = 2.2 MΩ	C_1_ = 10 µF	C_2_ = 100 µF
Comp1 = MAX934 Channel1	Comp1 = MAX934 Channel3	REF = T1 REF3312

**Table 2:** Power Loss Analysis in Boost Converter MPPT in 1 Duty Cycle (1 mH inductor; 14 µF input capacitor).

Total Input Power:	100%	500 µW
Loss in Inductor ESR:	10.6%	53 µW
Loss in Diode Forward Voltage Drop	0%	0 µW
Loss in MOSFET On-Resistance	2.8%	14 µW
Loss in SuperCap ESR	0.8%	4 µW
Loss in input capacitor ESR	0.5%	2.5 µW
Switching Loss:	0.8%	4 µW
**Total Output Power:**	**85.1%**	**425.5 µW**

**Table 3:** Sub 1 mW to 50 mW Input Power MPPT Results.

	Our Prototype	Tan [22]	Tan [23]	Chini [29]	Dondi [17]
**Year**	2015	2011	2012	2010	2008
**MPPT Converter**	Boost	Buck	Buck	Buck	Buck
**MPPT Control**	PWM FVOC	PFM FVOC	PFM FVOC	PFM FVOC	PWM FVOC
**Input Power**	0.5 mW	5 mW	0.4 mW	1.6 mW	50 mW
**Efficiency**	80.5%	47%	59%	30%	85%
